RETRACTED

# miR‐107 regulates growth and metastasis of gastric cancer cells via activation of the PI3K‐AKT signaling pathway by down‐regulating FAT4

**DOI:** 10.1002/cam4.2396

**Published:** 2019-07-12

**Authors:** Li Wang, Kunkun Li, Chen Wang, Xiaoxin Shi, Huiyu Yang

**Affiliations:** ^1^ Department of Gastroenterology Henan Provincial People's Hospital (Zhengzhou University People's Hospital Fuwai Central China Cardiovascular Hospital) Zhengzhou Henan Province China; ^2^ Department of Gastroenterology Zhengzhou Central Hospital Affiliated to Zhengzhou University Zhengzhou Henan Province China; ^3^ Department of Neck, Shoulder, Waist and Leg Zhengzhou Osteopathy Hospital Zhengzhou China; ^4^ Health Examination Centre Henan Provincial People's Hospital (Zhengzhou University People's Hospital Fuwai Central China Cardiovascular Hospital) Zhengzhou Henan Province China; ^5^ Department of Gastroenterology The First Affiliated Hospital of Zhengzhou University Zhengzhou Henan Province China

**Keywords:** FAT4, gastric cancer, metastasis, miR‐107, proliferation

## Abstract

**Purpose:**

To investigate the effect of miR‐107 on the growth and metastasis of gastric cancer (GC) and elucidate the probable mechanisms.

**Methods:**

The expression of miR‐107 and FAT4 in GC tissues and cells were detected using qRT‐PCR. Bioinformatics and dual luciferase reporter gene assays were used to analyze the relationship between miR‐107 and FAT4. miR‐NC, miR‐107 inhibitor, pcDNA3.1‐FAT4 and siRNA‐FAT4 were transfected into AGS and MKN‐45 GC cell lines, respectively. The proliferation and migration abilities of GC cells after transfection were evaluated using the MTT assay, scratch test and transwell assay. The expression of epithelial‐mesenchymal transition (EMT) markers: E‐cadherin, N‐cadherin, vimentin and related proteins of the PI3K/AKT signaling pathway were determined using western blot. The xenograft tumors of nude mice were observed to assess the tumorigenicity of GC cells in vivo.

**Results:**

MiR‐107 was up‐regulated, while FAT4 was down‐regulated in GC tissues and cells (*P* < 0.05); FAT4 was targeted and negatively regulated by miR‐107. Down‐regulating miR‐107 or up‐regulating FAT4 inhibited the GC cells proliferation, migration, invasion and tumorigenicity, and could also reduce the expression of N‐cadherin, vimentin, p‐PI3K and p‐Akt expression and up‐regulate E‐cadherin.

**Conclusions:**

miR‐107 promotes growth and metastasis in GC via activation of PI3K‐AKT signaling by targeting FAT4, which may be a target for GC treatment.

## 1 INTRODUCTION

Gastric cancer (GC) is one of the most common digestive malignancies.^1^ The global cancer statistics reports of the World Health Organization and the International Agency for Research on Cancer in 2018 reported that the death rate of GC ranked third among all malignant tumors worldwide.^2^ In China, both the morbidity and mortality of GC were obviously higher than western countries.^3^ The most important reasons of poor prognosis and death of malignant tumor including GC are reccurrence and metastasis. So sutdy on the molecular mechanism of the growth and metastasis of GC cells has important significance for the early diagnosis, treatment or prognosis of GC.

RETRACTED

More and more microRNAs (miRNAs) were reported as carcinogens or tumor suppressors, working with specific target genes to regulate the proliferation, metastasis or apoptosis of cancer cells including GC.^4^ MiRNA microarray had verified multiple miRNAs, containing miR‐107, were dysregulated in GC.^5^ miR‐107 had been proved to be a carcinogenic RNA in the development and progression of multiple cancers, such as in colorectal cancer by mediating Krüppel‐like factor4 (KLF4)^6^, ^7^ and in breast cancer by targeting Dicer.^8^ In GC, it was reported that miR‐107 as a carcinogen could promote invasion and migration by targeting Dicer1,^9^, ^10^ and the other reported miR‐107 could inhibit proliferation and invasion as tumor suppressors by down‐regulating CDK6.^11^, ^12^ Therefore, the role and molecular mechanisms of miR‐107 in GC remain controversial and need to be further studied.

FAT4 was first identified in a mouse mammary epithelial cell line, and played an important role in tumorigenesis and epithelial‐mesenchymal transition (EMT) in many cancers.^13^, ^14^ EMT was essential for the development and metastasis of cancers,^15^ and the PI3K/AKT signaling pathway was involved in the process.^16^ Currently, rare studies have explored the relationship between miR‐107 and FAT4, and their molecular mechanism in GC. In this study, FAT4 was first proposed to be a target gene of miR‐107, and the authors aimed to explore the effect of miR‐107 on the proliferation and migration of GC cells and the potential mechanism: it worked by targeting FAT4 via activation of the PI3K/AKT signaling pathway.

## 2 MATERIALS AND METHODS

### 2.1 Tissue specimens, cell and animals

Specimens of GC tissues and corresponding adjacent benign gastric mucosa were collected from 150 patients with GC, confirmed by pathological examination at the authors' hospital from January 2016 to January 2018. Inclusion criteria: (a) Primary GC; (b) No radiotherapy, chemotherapy or other therapy before surgery; (c) Without other primary tumors. The tissues were frozen and stored in liquid nitrogen. All patients had signed the informed consents.

Human gastric epithelial cell line (GES‐1), and GC cell lines KATO III, AGS, MGC‐803, MKN‐45, MKN‐28, HGC27 and NS‐3 were purchased from the American Type Culture Collection (ATCC, USA). All the cells were cultured in RPMI 1640 medium (Gibco, USA) with 10% fetal bovine serum (FBS, Gibco, USA), 1% penicillin (100 U/mL) and streptomycin (100 μg/mL) (Hyclone, USA) in an incubator with 5% CO_2_ and at 37°C.

80 BALB/c nude mice(6‐8 weeks, 20‐28g) were purchased from the Laboratory Animal Center of Zhenghzou University and fed on a standard diet and sterilized water to acclimate the environment for 7 days. Animal experiments adhered to the National Institutes of Health Guide for the Care and Use of Laboratory Animals and the study has been approved by the Ethics Committee of Henan Provincial People's Hospital.

RETRACTED

### 2.2 Dual luciferase reporter gene assay

miR‐107 could be complementary to the 3'‐UTR of FAT4 gene, which was predicted by the miRNAs target gene prediction database: TargetScan, miRDB and microRNA.org. The dual luciferase reporter gene assay was performed to verify the relationship between miR‐107 and FAT4. The special primers were designed according to the sequence of FAT4 gene (synthesized by Tsingke biological technology, Wuhan) to amplify the fragments of FAT4 3′‐UTR and FAT4 3′‐UTR mut containing miR‐107 binding site. Then the recombinant vectors Psi‐CHECK2‐FAT4‐3′‐UTR and Psi‐CHECK2‐FAT4‐3′‐UTR mut were constructed, screened and identified. Then the miR‐107 mimic or miR‐NC and Psi‐CHECK2‐FAT4‐3′‐UTR or Psi‐CHECK2‐FAT4‐3′‐UTR mut vector were transfected into 293T cells, respectively. After 48 hours of transfection, the luciferase activity was detected using dual luciferase reporter gene system (Promega, USA). The relative luciferase activity = Firefly fluorescence/Renilla fluorescence, with Renilla fluorescence as internal control.

### 2.3 Quantitative RT‐PCR (qRT‐PCR)

Total RNA was extracted using Trizol (Invitrogen, USA) according to the manufacturer's instructions. SuperScript First Strand cDNA reverse transcription kit was used to synthesize cDNA. RT‐PCR was performed using ABI7600 system (Applied Biosystems, USA) with special primers and SYBR Green PCR master mix. The reaction conditions were as follows: 95°C 10 minutes, and 40 cycles of 95°C 15 seconds, 60°C 15 seconds. The relative expression of miR‐107 and FAT4 were normalized to an endogenous reference control gene (RNU‐6B and β‐actin) and calculated using 2^−ΔΔCt^.

### 2.4 Cell transfection

Two kinds of cell lines with the highest miR‐107 expression were selected to proceed with the following experiments. miR‐NC, miR‐107 inhibitor, pc‐DNA3.1‐FAT4 plasmid, and siNA‐FAT4 were synthesized by Shanghai Sangon Biotech (Shanghai, China). The third passage of GC cells at the logarithmic phase were grouped into the blank control, miR‐NC group, miR‐107 inhibitor group, overexpression FAT4 group (pc‐DNA3.1‐FAT4 plasmid), miR‐107 inhibitor + siRNA‐FAT4 group. The cells were transfected according to the instructions of liporfectamine 2000 (Invitrogen, USA) when the cells at 50% fusion. After transfection for 6‐8 hours, the cells were replaced withnew medium for 24‐48 hours at 37°C with 5% CO_2_, for the following experiment.

RETRACTED

### 2.5 MTT assay

After transfection for 24 hours, the transfected cells were detached using 0.25% trypsin to seed into 96‐well plates (1 × 10^4^ cells/well).Ten microliters of MTT solution (5 mg/mL, Sigma, USA) was added and incubated for 4 hours in each well. Then 150 μL of DMSO (Sigma, USA) was added and shaken for 5 minutes for complete dissolution. Subsequently, the optical density (OD) value at 570 nm was detected using a microplate reader. The experiments were repeated three times. The cell proliferation curve was plotted with time point as the abscissa and OD value as the ordinate.

### 2.6 Cell wound scratch test

After transfection for 24 hours, cells that were in good condition were seeded into 6‐well plate (1 × 10^6^ cells/well) for culturing at 37°C, 5% CO_2._ A two hundred‐microliter‐pipette was used to create a wound, and the cells debris was removed using PBS when cells were at 80% fusion. Then the RPMI 1640 medium with 10% FBS was replaced with fresh serum‐free medium for culture. The scratch width as an indicator of migration distance was observed and photographed under a microscope at 0 and 24 hours. Experiments were repeated three times.

### 2.7 Transwell assay

The prepared matrigel (BD Biosciences, USA) was dissolved and diluted with medium in the apical chamber of an incubator. The transfected cells were suspended in the serum‐free RPMI 1640 medium to adjust the cell density to 1 × 10^5^. Two hundred microliters of cells were added in the upper chamber of 24‐well plate, and the RPMI 1640 medium with 10% FBS was placed in the lower chamber. After 24 hours, the invaded cells were fixed, stained with 0.1% crystal violet for 10 minutes and counted under a light microscope. Five visual fields were randomly selected for counting the numbers of invaded cells.

### 2.8 Western blot

Total protein of cells was extracted, and the concentrations were measured using BCA methods. The protein was separated using 10% SDS‐PAGE and transferred to polyvinylidene fluoride membrane (Millipore, Bedford, USA). The membrane was blocked for 1 hour in tris buffered saline tween with 5% skimmed milk. Then the primary antibodies (Abcam, USA): FAT4 (1:500), E‐cadherin (1:1000), N‐cadherin (1:2000), vimentin (1:1000), PI3K (1:2000), AKT (1:5000), p‐AKT (1:3000), β‐actin (1:5000) were incubated at 4°C overnight. The specific secondary antibodies were incubated for 1 hour. The protein bands were observed using electrochemiluminescence detection reagent. The band densities were calculated using Image J software with β‐actin as internal reference.

RETRACTED

### 2.9 Xenograft tumor in nude mice

The mice were divided into five groups: blank control, miR‐NC, miR‐107 inhibitor, overexpression FAT4 and miR‐107 inhibitor + siRNA‐FAT4 groups. The transfected GC cell density was adjusted to 1 × 10^7^ cells/mL with PBS. The 200 μL‐cell suspension was subcutaneously injected into nude mice in each group. The survival status of each nude mice was observed and the maximum and minimum diameter (a and b) of implanted tumor in mice was measured with a vernier caliper once every 2 days. Tumor volume was calculated using the formula: Volume (mm^3^) = (a × b^2^)/2. The tumor was isolated when mice were sacrificed after 28 days.

### 2.10 Statistical analysis

All data were analyzed by SPSS19.0 software. Kolmogorov‐Smirnov(K‐S) test was used to detec if the data obey normal distribution. Measurement data were presented as mean ± standard deviation. One way analysis of variance was used to assess the comparison among multiple groups, while comparison between two groups were detected using the *t* test. The enumeration data were analyzed using χ^2^. *P* < 0.05, represented statistically significant difference.

## 3 RESULTS

### 3.1 FAT4 was a target gene of miR‐107

The target gene prediction database predicted that FAT4 might be targeted by miR‐107, as a result of the specific binding site between FAT4 3′‐UTR and miR‐107. The dual luciferase reporter gene assay was applied to verify if miR‐107 directly targeted FAT4. Compared with the NC groups, the relative luciferase activity of Psi‐CHECK2‐FAT4‐3′‐UTR was inhibited by miR‐107, while that of Psi‐CHECK2‐FAT4‐3′‐UTR mut did not have effect (Figure 1A). The results indicated that miR‐107 might specifically bind to FAT4.

**Figure 1:** Luciferase assay and the expression of miR‐107 and FAT4 in the transfected cells. A, The predicted relationship between miR‐107 and FAT4 using bioinformatics prediction website and dual luciferase reporter gene assay, *P < 0.05 vs miR‐NC; B, Relative expression of miR‐107 in transfected cells; C, Relative expression of FAT4 protein in transfected cells; 1, 2, 3, 4, 5 represented blank, miR‐NC, miR‐107 inhibitor, overexpression FAT4, miR‐107 inhibitor + siRNA FAT4 groups, respectively; D, Relative expression of FAT4 mRNA in transfected cells, *P < 0.05 vs blank and miR‐NC groups

RT‐PCR and Western blot were performed to determine miR‐107 and FAT4 expression in the cells following transfection to verify the regulated effect of miR‐107 on FAT4 (Figure 1B‐D). Compared to the blank and miR‐NC groups, the expression of miR‐107 decreased, and the mRNA and protein level of FAT4 increased in the miR‐107 inhibitor group, with significant difference. There was no difference in miR‐107 expression among the blank, miR‐NC and over‐expression FAT4 groups, while the FAT4 expression in the overexpression FAT4 group was higher than the blank and miR‐NC groups. No difference in FAT4 expression was found among blank, miR‐NC and miR‐107 inhibitor + siRNA‐FAT4 groups. The findings indicated that miR‐107 might negatively regulate FAT4.

RETRACTED

### 3.2 The expression of miR‐107 and FAT4 in GC tissues and cells

The expression of miR‐107 in GC tissues was significantly higher, while the expression of FAT4 mRNA was lower than that in adjacent normal tissues (*P* < 0.05) (Figure 2A and B). miR‐107 expression was negatively associated with FAT4 in GC tissues (*r* = −0.362, *P* < 0.001).

**Figure 2:** Expression of miR‐107 and FAT4 mRNA in GC tissues and cell lines and cell proliferation following transfection. A, Expression of miR‐107 in GC tissues; B, Expression of FAT4 mRNA in GC tissues; C, Expression of miR‐107 in GC cells; D, Expression of FAT4 mRNA in GC cells; **P < 0.01 vs GES‐1 cell. E and F, Cell proliferation ability curves of AGS cells and MKN‐45 cells; *P < 0.05 vs blank and miR‐NC groups

Compared with GES‐1, the expression of miR‐107 in KATO III, AGS, MGC‐803, MKN‐45, MKN‐28, HGC27 and NS‐3 cells was up‐regulated, while the expression of FAT4 was down‐regulated, especially in **AGS** and **MKN‐45** cells and they were selected to proceed with the following experiments (Figure 2C and D).

### 3.3 Down‐regulation of miR‐107 or up‐regulation of FAT4 inhibited GC cells proliferation

The MTT assay was performed to detect the proliferation ability of AGS and MKN‐45 cells following transfection (in Figure 2E and F). There was no difference in cell proliferation ability at 24 hours among all groups. The cell proliferation ability was obviously weaker in the miR‐107 inhibitor and overexpression FAT4 groups than that in the blank and miR‐NC groups at 48 and 72 hours (*P* < 0.05). Cell proliferation ability in the miR‐107 inhibitor + siRNA‐FAT4 group was higher than in the miR‐107 inhibitor group, while no difference in cell proliferation ability was found among the blank, miR‐NC and miR‐107 inhibitor + siRNA‐FAT4 groups at 48 and 72 hours. The results demonstrated that the proliferation of AGS and MKN‐45 GC cells was inhibited after transfection with miR‐107 inhibitor or over‐expression FAT4 vector.

RETRACTED

### 3.4 Down‐regulation of miR‐107 or up‐regulation of FAT4 inhibited GC cells migration and invasion

Scratch test was used to assess the cell migration (Figure 3). The cell migration distance in miR‐107 inhibitor and over‐expression FAT4 groups was found to be shorter than the blank and miR‐NC groups after culturing for 24 hours (*P* < 0.05), while no difference was found among the blank, miR‐NC and miR‐107 inhibitor + siRNA‐FAT4 groups (*P* > 0.05). The results suggested that down‐regulation of miR‐107 or up‐regulation of FAT4 might inhibit GC cells migration.

**Figure 3:** Cell migration was detected using scratch test. A, AGS cells migration following transfection; B, MKN‐45 cells migration following transfection. *P < 0.05 vs the blank and miR‐NC groups

The cell invasion was detected using transwell assay (Figure 4). The cell invasion abilities were weaker in the miR‐107 inhibitor and overexpression FAT4 groups than in the blank and miR‐NC groups (*P* < 0.05), while no difference was observed among the blank, miR‐NC and miR‐107 inhibitor + siRNA‐FAT4 groups (*P* > 0.05). All results suggested that down‐regulation of miR‐107 or up‐regulation of FAT4 inhibited the invasion of AGS and MKN‐45 GC cells.

**Figure 4:** Cells invasion was assessed using transwell assay. A, AGS cells invasion following transfection; B, MKN‐45 cells invasion following transfection. *P < 0.05 vs the blank and miR‐NC groups

### 3.5 Down‐regulation of miR‐107 or up‐regulation of FAT4 inhibited GC cells EMT

Western blot was conducted to detect the expression of EMT markers: E‐cadherin, N‐cadherin and vimentin.^17^ The results (Figure 5) demonstrated that, compared with the levels in blank and miR‐NC groups, FAT4 and E‐cadherin expression increased, while N‐cadherin and vimentin expression decreased in miR‐107 inhibitor and over‐expression FAT4 groups (*P* < 0.05). In contrast, FAT4 and E‐cadherin expressions were reduced, while N‐cadherin and vimentin expressions increased in miR‐107 inhibitor + siRNA‐FAT4 group. No significant difference was observed among the blank, miR‐NC and miR‐107 inhibitor + siRNA‐FAT4 groups. The results presented above indicate that down‐regulation of miR‐107 or up‐regulation of FAT4 inhibited EMT of AGS and MKN‐45 GC cells, further inhibiting the migration and invasion.

**Figure 5:** miR‐107 inhibitor and FAT4 inhibited the EMT. A, Protein bands and protein level of FAT4, E‐cadherin, N‐cadherin and vimentin in AGS cells following transfection were measured using Western blot analysis. B, Protein bands and protein level of FAT4, E‐cadherin, N‐cadherin and vimentin in MKN‐45 cells following transfection were measured using Western blot analysis. *P < 0.05 vs the blank and miR‐NC groups

RETRACTED

### 3.6 Down‐regulation of miR‐107 or up‐regulation of FAT4 inhibited the PI3K‐AKT signaling pathway

Proteins related to the PI3K‐AKT pathway were determined to explore whether the effect of miR‐107 or FAT4 on the GC cells was related to the PI3K‐AKT signal pathway (Figure 6). There was no difference in PI3K and AKT expression among all groups (*P* > 0.05). Compared with the blank and miR‐NC groups, the expression of p‐PI3K and p‐AKT obviously decreased in the miR‐107 inhibitor and overexpression FAT4 groups (*P* < 0.05). Compared with miR‐107 inhibitor group, the expression of p‐AKT and p‐PI3K increased, with significant difference (*P* < 0.05). The results suggested that down‐regulation of miR‐107 or up‐regulation of FAT4 inhibited the activation of the PI3K‐AKT signaling pathway.

**Figure 6:** miR‐107 inhibitor and FAT4 suppressed the PI3K‐AKT signaling pathway in GC cells. A, Protein bands and protein level of PI3K, p‐PI3K, AKT and p‐AKT in AGS cells following transfection were measured using Western blot analysis. B, Protein bands and protein lel of PI3K, p‐PI3K, AKT and p‐AKT in MKN‐45 cells following transfection were measured using Western blot analysis. *P < 0.05 vs the blank and miR‐NC groups

### 3.7 Down‐regulation of miR‐107 or up‐regulation of FAT4 suppressed tumorigenicity

Xenograft tumor in nude mice was detected to assess the cell tumorigenicity following transfection: 4 days after inoculation, the tumor volume was detected every 4 days and the tumor volume growth curve is shown in Figure 7. Compared with the blank and miR‐NC groups, the tumor growth were slow and the tumor volumewere reduced from the 12d in miR‐107 inhibitor and overexpression FAT4 groups (*P* < 0.05), while no obvious changes were detected in the miR‐107 inhibitor+siRNA‐FAT4 group (*P* > 0.05). The results demonstrated that down‐regulation of miR‐107 or up‐regulation of FAT4 suppressed the growth of xenograft tumors.

**Figure 7:** Tumor volume in nude mice injected with GC cells. A, Tumor growth curves following injection in AGS cells; B, Tumor growth curves following injection in MKN‐45 cells. *P < 0.05 vs the blank and miR‐NC groups

## 4 DISCUSSION

In recent years, miRNAs, as carcinogens or tumor suppressors, have involved in the development, invasion and metastasis of tumor by inhibiting the target gene expression. Multiple studies have shown that miR‐107 plays a crucial role in the development and metastasis of cancers. However, it was worth noting that miR‐107 had different or contradictory roles in different cancers. For example, miR‐107 could function as a tumor suppressor gene in esophageal carcinoma,^18^ lung cancer^19^ and hepatocellular carcinoma,^20^ whereas act as an oncogene in liver cancer^21^ and colorectal cancer.^6^ However, studies have shown that miR‐107 may play different or even opposite roles in the same cancer. Zhang et al^22^ found that miR‐107 targeted down‐regulating Siah1, promoted proliferation, migration and invasion, and inhibited apoptosis in human breast cancer cell, while Gao et al^23^ revealed that miR‐107 was down‐regulated in breast cancer tissue and cell lines, and could markedly suppress proliferation, cell cycle progression and invasion of breast cancer cell by inhibiting the expression of BDNF. In GC, Feng et al^11^ found that miR‐107 might be a tumor suppressor, which inhibited the proliferation and invasion by directly targeting CDK6 in GC cells. Cheng et al^24^ also indicated that miR‐107 was a tumor inhibitor that down‐regulated BDNF expression and inactivated the PI3K/AKT signaling pathway to inhibit the proliferation and metastasis of GC. However, Li et al^25^ reported an opposite role that miR‐107 was up‐regulated in GC tissues and promoted GC cell proliferation by negatively targeting FOXO1; Song et al^26^ identified that as an oncogene, miR‐107 promoted proliferation of GC by regulating CDK8; Wang et al^27^ also indicated that miR‐107 was up‐regulated in GC, and suppressed the proliferation and invasion by negatively regulating NF1 expression. In this study, the authors found that miR‐107 was up‐regulated both in GC tissues and cells, consistent with the results of part present researches.^25^, ^26^, ^27^, ^28^ Down‐regulating miR‐107 could inhibit the proliferation, migration and invasion of GC cells and reduced the tumorigenicity in nude mice, meaning miR‐107 may serve as an oncogene in GC.

RETRACTED

FAT4 was shown to act as a tumor suppressor, involving in the development and metastasis of tumors. In this study, target gene prediction and dual luciferase report gene assay results verified that FAT4 was the downstream gene of miR‐107 and FAT4 was regulated negatively by miR‐107. In addition, up‐regulating FAT4 could inhibit the GC cells proliferation and suppress the growth of xenograft tumor in nude mice, which was similar to the results of down‐regulating miR‐107. Cai et al^29^ demonstrated that down‐regulation of FAT4 could promote the growth, EMT of GC cells via activation of Wnt/β‐actin signaling. EMT is an vital mechanism of tumor cell invasion and metastasis, with the declining of E‐cadherin and increasing of N‐cadherin, vimentin in its process.^30^ In this study, E‐cadherin was increased and N‐cadherin and vimentin was reduced after down‐regulating miR‐107 or up‐regulating FAT4, demonstrating that miR‐107 and FAT4 may affect the migration and invasion of GC cells by regulating EMT, which was consistent with this study. Multiple studies had indicated that PI3K/AKT signaling was involved in regulating the proliferation, apoptosis and metastasis of GC or other tumors by inducing EMT.^31^, ^32^ Wei et al^33^ indicated that FAT4 could promote autophagy and inhibit the EMT of colorectal cancer, by regulating the PI3K/AKT/mTOR and PI3K/AKT/GSK‐3β signaling pathway. To further explore whether FAT4 inhibited the EMT of GC cells by regulating PI3K/AKT, the related protein of PI3K/AKT signaling was detected using Western blotting in this study. Down‐regulation miR‐107 or up‐regulation FAT4 could decrease p‐PI3K and p‐AKT expression, indicating that up‐regulating FAT4 could inhibit the proliferation, migration and invasion of GC cells by inactivating the PI3K/AKT signaling pathway.

## 5 CONCLUSIONS

In summary, the study demonstrated that miR‐107, as an oncogene, was up‐regulated in GC tissues and cells. miR‐107 could promote the proliferation, migration and invasion of GC cells by targeting FAT4. The mechanism of miR‐107 promoted the proliferation and metastasis of GC was promoted the EMT tand the activation of PI3K/AKT signaling pathway by targeting FAT4. The study may provide a new biological marker miR‐107 to predict the progress and prognosis of GC, and lay a theoretical foundation to some extent for the study of the development, especially for the invasion and metastasis of GC.

## CONFLICT OF INTERESTS

All authors declare no conflict of interest, financial or otherwise.
